The article "SP1-induced lncRNA AGAP2-AS1 expression promotes chemoresistance of breast cancer by epigenetic regulation of MyD88" was retracted in 2023. Reasons: duplicated images; signs of a paper mill; unreliable results or conclusions.

# SP1-induced lncRNA AGAP2-AS1 expression promotes chemoresistance of breast cancer by epigenetic regulation of MyD88

**DOI:** 10.1186/s13046-018-0875-3

**Published:** 2018-08-29

**Authors:** Huaying Dong, Wei Wang, Shaowei Mo, Ru Chen, Kejian Zou, Jing Han, Fan Zhang, Jianguo Hu

**Affiliations:** 1 Department of General Surgery, Hainan General Hospital, Jinan University, No.19 Xiu Hua Road, Xiuying District, Haikou city, 570311 Hainan Province China; 2 Department of Science and Education, Hainan Maternal and Child health hospital, Haikou, 570206 Hainan China; 3 Department of Obstetrics and Gynecology, The Second Affiliated Hospital, Chongqing Medical University, Chongqing, 400010 China

**Keywords:** SP1, Breast cancer, lncRNA AGAP2-AS1, MyD88, H3K27 acetylation, Trastuzumab

## Abstract

**Background:**

Resistance to trastuzumab has become a leading cause of mortality in breast cancer patients and is one of the major obstacles for improving the clinical outcome. Cell behavior can be modulated by long non-coding RNAs (lncRNAs), but the contribution of lncRNAs in trastuzumab resistance to breast cancer is largely unknown. To this end, the involvement and regulatory function of lncRNA AGAP2-AS1 in human breast cancer are yet to be investigated.

**Methods:**

Trastuzumab-resistant SKBR-3 and BT474 cells were obtained by continuous culture with 5 mg/mL trastuzumab for 6 months. RT-qPCR assay was used to determine the expression of AGAP2-AS1 in tissues and cells. RNA fluorescence in situ hybridization was used to investigate the subcellular location of AGAP2-AS1 in breast cancer cells. Bioinformatic analysis, chromatin immunoprecipitation (ChIP), RNA immunoprecipitation (RIP), western blotting, and immunofluorescence were carried out to verify the regulatory interaction of AGAP2-AS1, CREB-binding protein (CBP), and MyD88. In addition, a series of in vitro assays and a xenograft tumor model were used to analyze the functions of AGAP2-AS1 in breast cancer cells.

**Results:**

AGAP2-AS1 was upregulated and transcriptionally induced by SP1 in breast cancer. Overexpression of AGAP2-AS1 promoted cell growth, suppressed apoptosis, and caused trastuzumab resistance, whereas knockdown of AGAP2-AS1 showed an opposite effect. MyD88 was identified as a downstream target of AGAP2-AS1 and mediated the AGAP2-AS1-induced oncogenic effects. Mechanistically, the RIP assay revealed that AGAP2-AS1 could bind to CBP, a transcriptional co-activator. ChIP assays showed that AGAP2-AS1-bound CBP increased the enrichment of H3K27ac at the promoter region of MyD88, thus resulting in the upregulation of MyD88. Gain- and loss-of-function assays confirmed that the NF-κB pathway was activated by MyD88 and AGAP2-AS1. Furthermore, high AGAP2-AS1 expression was associated with poor clinical response to trastuzumab therapy in breast cancer patients.

The article "SP1-induced lncRNA AGAP2-AS1 expression promotes chemoresistance of breast cancer by epigenetic regulation of MyD88" was retracted in 2023. Reasons: duplicated images; signs of a paper mill; unreliable results or conclusions.

**Conclusion:**

AGAP2-AS1 could promote breast cancer growth and trastuzumab resistance by activating the NF-κB signaling pathway and upregulating MyD88 expression. Therefore, AGAP2-AS1 may serve as a novel biomarker for prognosis and act as a therapeutic target for the trastuzumab treatment.

**Electronic supplementary material:**

The online version of this article (10.1186/s13046-018-0875-3) contains supplementary material, which is available to authorized users.

## Background

Breast cancer has become a leading cause of cancer-related deaths worldwide and is the most common cancer among women [1]. The important reason for these deaths is distant metastasis and resistance to the currently available therapeutics [2]. About 15–20% of breast cancer patients showing an overexpression of human epidermal growth factor receptor 2 (HER2) demonstrate poorer prognosis and survival [3, 4]. Currently, therapies with anti-HER2 monoclonal antibody such as trastuzumab are administered to treat HER2-positive breast cancer patients [5, 6]. Trastuzumab is designed to target HER2 and silence its function. It is mostly administered to patients with early-stage or metastatic gastric and breast cancer with positive HER2 mutations. However, the initial positive effects of trastuzumab gradually decrease owing to the increased resistance after exposure. In addition, there is a clear need for the development of a useful therapeutic biomarker for predicting chemoresponse to trastuzumab treatment [7].

With the advancements in whole genome and transcriptome sequencing technologies and the ENCODE project, it has become clearer that most of the genomic DNA is represented as processed transcripts lacking the protein-coding ability [8]. Long non-coding RNAs (lncRNAs) are a recently discovered major class of non-coding RNAs (ncRNAs) that have a length of more than 200 nucleotides [9]. In recent years, emerging evidence has indicated that some lncRNAs such as AGAP2-AS1 play an important role in regulating gene expression and biological functions through epigenetic regulation, including methylation, acetylation, and ubiquitination [10–12].

AGAP2-AS1, which is transcribed from a gene located on 12q14.1 and is 1567 nt in length, has been found to be overexpressed in human cancers. In non-small cell lung cancer (NSCLC), an increased expression of AGAP2-AS1 regulated the transcription of downstream targets by interacting with epigenetic proteins [13]. Myeloid differentiation factor 88 (MyD88) is defined as a carcinogenic protein, promoting tumor growth and metastasis, which make it a prognostic and therapeutic target [14]. Previously, Xu et al. demonstrated that MyD88 was epigenetically regulated by H3K27 modifications in hepatocellular carcinoma [15]. However, the role of AGAP2-AS1 in trastuzumab resistance and the interaction between AGAP2-AS1 and MyD88 are not well known.

The article "SP1-induced lncRNA AGAP2-AS1 expression promotes chemoresistance of breast cancer by epigenetic regulation of MyD88" was retracted in 2023. Reasons: duplicated images; signs of a paper mill; unreliable results or conclusions.

In this study, we hypothesized that lncRNA AGAP2-AS1 affects breast cancer growth and resistance via regulating MyD88 expression through H3K27 acetylation. To verify this hypothesis, we determined the expression level of AGAP2-AS1 in breast cancer tissues and cell lines. By performing in vitro and in vivo experimental assays, we further investigated the functional relevance of AGAP2-AS1 in breast cancer chemoresistance.

## Methods

### Patient samples

Primary cancer tissue and adjacent noncancerous tissue samples were collected from a cohort of 42 patients with breast cancer (male/female: 0/42, range of age (median): 38–61 (47)), and another independent cohort of 67 HER2^+^ breast cancer patients who received trastuzumab treatment (male/female: 0/67, range of age (median): 47–82 (55)). The diagnoses of all the patients were pathologically confirmed, and the clinical tissue samples were collected before chemotherapy was started at Hainan General Hospital and The Second Affiliated Hospital of Chongqing Medical University. The samples were obtained during operation and immediately frozen at − 80 °C until RNA extraction. The written informed consents obtained from all patients were approved according to the guidelines revised by the Hainan General Hospital.

### Cell lines and reagents

The human breast cancer cell lines SKBR-3 and BT474, which harbor HER2-activating mutations, were purchased from Chinese Type Culture Collection, Chinese Academy of Sciences (Shanghai, China). Both the cell lines were cultured in DMEM (BioWhittaker, Lonza, USA) supplemented with 1 mM L-glutamine, 100 U/ml penicillin/streptomycin (BioWittaker, Lonza) and heat-inactivated 10% fetal bovine serum (FBS, Gibco) at 37 °C in a humidified incubator with 5% CO_2_. Trastuzumab (Herceptin) was obtained from Roche (Basel, Switzerland) and dissolved in the enclosed sterile water. The trastuzumab-resistant SKBR-3/Tr and BT474/Tr cells were obtained by continuous culture with 5 μg/mL trastuzumab for 6 months as previously reported [16–18].

### RNA oligoribonucleotides and cell transfection

The full-length of lncRNA AGAP2-AS1, and the coding sequence of MyD88 and CREB-binding protein (CBP) were amplified and cloned into the lentivirus vector (Lv-AGAP2-AS1, Lv-MyD88, and Lv-CBP, respectively) for retrovirus production using BT474 cells by GeneChem (Shanghai, China). The negative control vectors were also generated. The lentivirus vector containing small hairpin RNA (shRNA) sequence targeting MyD88 (sh-MyD88), AGAP2-AS1 (sh-AGAP2-AS1) or negative control vector (sh-NC) was also amplified and cloned by GeneChem. All the vectors were labeled with green fluorescence protein (GFP). Transfection was carried out using Lipofectamine 3000 (Invitrogen, Carlsbad, CA, USA) following the manufacturer’s instructions. Transfection efficiency was evaluated in every experiment by RT-qPCR after 24 h to ensure that cells were transfected. Functional experiments were then performed after sufficient transfection for 48 h. The sequences of shRNAs are shown in the Additional file 1: Table S1.

The article "SP1-induced lncRNA AGAP2-AS1 expression promotes chemoresistance of breast cancer by epigenetic regulation of MyD88" was retracted in 2023. Reasons: duplicated images; signs of a paper mill; unreliable results or conclusions.

### Reverse transcription-quantitative polymerase chain reaction (RT-qPCR)

The RNA was reverse transcribed using the SuperScript III® (Invitrogen) and then the obtained cDNAs were quantified using RT-qPCR assay labeled with SYBR (Takara Bio Company, Dalian, China) on BioRad CFX96 Sequence Detection System (BioRad company, Berkeley, CA). The gene expression levels were normalized using GAPDH expression. The RT-qPCR results were analyzed and expressed relative to the CT (threshold cycle) values, and then converted to fold changes. All the primer sequences were synthesized by RiboBio (Guangzhou, China), and their sequences are shown in Additional file 1: Table S1.

### Cell viability assay

The altered cell viability after transfection was assayed using the MTT Kit (Dojindo, Rockville, MD, USA). In brief, cells were seeded into a 96-well plate and then treated with silencing or overexpressing vectors for 48 h. Next, the cells were treated with the MTT reagent and further cultured for 2 h. The optical density at 450 nm was measured with a spectrophotometer (Thermo Electron Corporation, MA, USA). The percentage of the control samples for each cell line was calculated thereafter.

### Chromatin immunoprecipitation (ChIP) and RNA immunoprecipitation (RIP)

ChIP was performed using the EZ ChIP™ Chromatin Immunoprecipitation Kit (Millipore, Burlington, MA) according to the manufacturer’s protocol. Briefly, cross-linked chromatin was sonicated into 200–1000 bp fragments. The chromatin was immunoprecipitated using anti-H3K27ac (Abcam, ab4729, Cambridge, MA)and anti-CBP antibodies (Abcam, ab2832). Magna RIP™ RNA-Binding Protein Immunoprecipitation Kit (Millipore) was used for RIP and anti-CBP antibody was used to pull down AGAP2-AS1.

### Immunofluorescence

The cells were fixed in 4% formaldehyde for 15 min and then washed with PBS. The fixed cells were then treated with pepsin and dehydrated through ethanol, and further permeabilized in Triton X100 (Sigma-Aldrich) for 20 min. Goat serum was used for blocking, and then cells were incubated with the anti-Ki67 antibody (Abcam, ab15580, 1:500, Cambridge, MA) overnight at 4 °C. The primary antibody was washed off, and then the cells were incubated with the appropriate rhodamine-conjugated secondary antibody for 1 h. The cells were again washed and incubated with DAPI (Invitrogen) for nuclear staining. The cells were visualized for immunofluorescence with a fluorescence microscope (DMI4000B, Leica).

The article "SP1-induced lncRNA AGAP2-AS1 expression promotes chemoresistance of breast cancer by epigenetic regulation of MyD88" was retracted in 2023. Reasons: duplicated images; signs of a paper mill; unreliable results or conclusions.

### Fluorescence in situ hybridization analysis (FISH)

The nuclear and cytosolic fraction separation was performed using the PARIS kit (Life Technologies), and RNA FISH probes were designed and synthesized according to the manufacturer’s instructions. Briefly, cells were fixed in 4% formaldehyde for 15 min and then washed with PBS. The fixed cells were treated with pepsin and dehydrated through ethanol. The air-dried cells were incubated further with 40 nM of the FISH probe in hybridization buffer (Life Technologies). After hybridization, the slide was washed, dehydrated and mounted with Prolong Gold Antifade Reagent with DAPI for detection. The slides were visualized for immunofluorescence with a fluorescence microscope (DMI4000B, Leica).

### TUNEL assay

The TUNEL staining was performed to evaluate cell apoptosis. In brief, cells were fixed by using 4% formaldehyde followed by staining with the TUNEL kit according to the manufacturer’s instructions (Vazyme, TUNEL Bright-Red Apoptosis Detection Kit, A113). The TUNEL-positive cells were counted under the fluorescence microscope (DMI4000B, Leica).

### In vivo mice xenograft assay

Male BALB/C nude mice (6 weeks of age) were purchased from Shanghai SIPPR-BK Laboratory Animal Co. Ltd. (Shanghai, China) and maintained in microisolator cages. Mice were housed in a facility-controlled, pathogen-free conditions under 28 °C, 50% humidity and were fed ad libitum with sterile chow food and water. All efforts were made to minimize suffering and the research protocol was approved by Hainan General Hospital of Jinan University based on Ethics in the Care and Use of Laboratory Animals. 1 × 10^7^ BT474 cells stably transfected with Lv-NC/Lv-AGAP2-AS1, or co-transfected with sh-MyD88/sh-NC and Lv-AGAP2-AS1 were suspended in 110 μL of serum-free DMEM, and then injected subcutaneously in the flank. When tumors were palpable, mice were treated by administering 5 mg/kg trastuzumab or PBS (in case of control) intraperitoneally once every 2 days for 3 weeks. Herein, six mice xenograft treatment groups were established: (Lv-NC-transfected cells + PBS, (Lv-AGAP2-AS1-transfected cells + PBS), (Lv-NC-transfected cells + trastuzumab treatment), (Lv-AGAP2-AS1-transfected cells + trastuzumab treatment), (Lv-AGAP2-AS1/sh-NC-cotransfected cells + trastuzumab treatment) and (Lv-AGAP2-AS1/sh-MyD88-cotransfected cells + trastuzumab treatment). Six mice were included in each group and more than three mice remained at the end of the study, excluding mice that were dead or had complications, such as skin necrosis due to infection. At the end of the treatment that lasts for 3 weeks, the xenograft tumor was stripped, and the mass was calculated. The tumor size was evaluated using a standard caliper measuring tumor length and width in a blinded manner and the tumor volume was calculated using the formula: length × width^2^ × 0.52.

The article "SP1-induced lncRNA AGAP2-AS1 expression promotes chemoresistance of breast cancer by epigenetic regulation of MyD88" was retracted in 2023. Reasons: duplicated images; signs of a paper mill; unreliable results or conclusions.

### Immunohistochemistry (IHC) analysis

Immunohistochemical staining was performed on 4-μm-thick sections. Briefly, the slides were deparaffinized and antigen retrieval was performed in a steam cooker for 1.5 min in 1 mM EDTA. Rabbit anti-MyD88 antibody (Abcam, ab2064) at 1:150 dilution was added and incubated overnight at 4 °C. The universal secondary antibody (DAKO) was applied for 15 min at room temperature. Diaminobenzidine or 3-amino-9-ethylcarbazole was used as chromogens and slides were counterstained with hematoxylin before mounting.

### Western blots and antibodies

The cell lysates were prepared with RIPA buffer containing protease inhibitors (Sigma-Aldrich). The membranes were incubated overnight at 4 °C with of the primary antibodies at a dilution of 1:1000. A secondary antibody was then used for immunostaining for 1 h at room temperature. The primary antibodies used in this study are anti-MyD88 (Abcam, ab2064), anti-CBP (Abcam, ab50702), anti-SP1 (Abcam, ab124804) anti-NF-κB p65 (Abcam, ab16502), and anti-β-actin (Abcam, ab6276) antibody.

### Statistical analysis

All the measurement data are represented as the median value. The count dates were described as frequency and examined using Fisher’s exact test. The Mann-Whitney U test or Kruskal-Wallis test was used for evaluating the difference among different clinical or cell-treated groups. Spearman correlation test was performed to identify the correlation between MyD88 and AGAP2-AS1. Receiver Operating Characteristic (ROC) curve was used to discriminate responders and non-responders to trastuzumab therapy. All statistical analyses were performed with SPSS 17.0 software (SPSS Incorporation, Chicago, IL). Error bars in figures represent SD (standard deviation). The results were considered statistically significant if *p* < 0.05.

## Results

### LncRNA AGAP2-AS1 is induced by SP1 in breast cancer cells

The RT-qPCR analysis was performed to detect the expression of AGAP2-AS1 in the breast cancer cells. As shown in Fig. 1a, AGAP2-AS1 was upregulated in the breast cancer cell lines when compared to the normal breast epithelium MCF-10A cells. To investigate whether AGAP2-AS1 regulates trastuzumab resistance, we established two trastuzumab-resistant sub-lines derived from HER2^+^ SKBR-3 and BT474 cells (SKBR-3/Tr and BT474/Tr, respectively). Compared with the parental cells, the established resistant cells showed less response to trastuzumab treatment, as evidenced by increased IC_50_ values and elevated cell viability (Fig. 1b, c). Moreover, AGAP2-AS1 was upregulated in trastuzumab-resistant cells than in the respective parental cells (Fig. 1d). This indicates that AGAP2-AS1 may be critical for breast cancer progression.

The article "SP1-induced lncRNA AGAP2-AS1 expression promotes chemoresistance of breast cancer by epigenetic regulation of MyD88" was retracted in 2023. Reasons: duplicated images; signs of a paper mill; unreliable results or conclusions.

**Fig. 1:** LncRNA AGAP2-AS1 is upregulated and induced by SP1 in breast cancer cells. **a** RT-qPCR was performed to detect the expression level of AGAP2-AS1 in breast cancer cells. **b** The IC_50_ value of trastuzumab was detected for both sensitive and resistant cells by cell viability assay. **c** The cell viability of both trastuzumab-resistant and sensitive cells were determined. **d** AGAP2-AS1 expression was identified by RT-qPCR in both trastuzumab-resistant and sensitive cells. **e** Prediction of SP1 binding site in the AGAP2-AS1 promoter region using JASPAR (http://jaspar.genereg.net/). **f** The expression of SP1 in gefitinib resistant and parental cells at transcript (left panel) and protein (right panel) levels. **g** RT-qPCR analysis of AGAP2-AS1 expression after SP1 was overexpressed. **h** FISH analysis of the enriched level of SP1 gene in nucleus of the SKBR-3 or SKBR-3/Tr cells. **i** ChIP assay was performed to detect the relative enrichment of SP1 in promoter of AGAP2-AS1. **j** Schematic presentation of SP1 binding sites in the promoter region of AGAP2-AS1. **k** Luciferase activity analysis of the two binding sites in cells transfected with respective oligonucleotides. *p < 0.05, **p < 0.01, ***p < 0.001

There have been evidence indicating that transcription factors (TFs) play an important role in lncRNA dysregulation, and hence, we searched for transcription factors that might be linked to lncRNA dysregulation. By using the online transcription factor prediction software JASPAR (http://jaspar.genereg.net/), we found that there are 11 SP1 binding sites in the promoter region of AGAP2-AS1 (Fig. 1e). Previously, Qi et al. demonstrated that AGAP2-AS1 is activated by SP1 in gastric cancer [19]. Therefore, we investigated whether this interaction also applies to breast cancer. We identified that SP1 was upregulated in the trastuzumab-resistant cells when compared to the parental cells at both transcript and protein levels (Fig. 1f). Transfection of SP1-overexpression vector dramatically increased AGAP2-AS1 expression levels (Fig. 1g). Consistently, the immunofluorescence assay showed that SP1 enrichment significantly increased in the nucleus of the SKBR-3 resistant cells when compared to the parental cells (Fig. 1h). We also performed ChIP assay to further verify the enrichment of SP1 at the promoter region of AGAP2-AS1. As expected, SP1 was enriched and the enrichment significantly increased in the resistant cells in contrast to the parental cells (Fig. 1i). In addition, the AGAP2-AS1 promoter region including 2 binding sites of SP1 with a high score was inserted into a PGL3 vector (Fig. 1j), and dual-luciferase reporter assay indicated that SP1 significantly promoted the luciferase activity (Fig. 1k). These results indicated that the upregulation of AGAP2-AS1 in breast cancer cells may be induced by SP1.

The article "SP1-induced lncRNA AGAP2-AS1 expression promotes chemoresistance of breast cancer by epigenetic regulation of MyD88" was retracted in 2023. Reasons: duplicated images; signs of a paper mill; unreliable results or conclusions.

### lncRNA AGAP2-AS1 promotes cell growth and inhibits apoptosis in breast cancer

Next, we investigated the functional role of AGAP2-AS1 in proliferation and apoptosis of breast cancer cell lines. The expression studies revealed that endogenous expression of AGAP2-AS1 in SKBR-3 breast cancer cell line was high while BT474 showed a low endogenous expression. Therefore, we constructed the AGAP2-AS1 overexpression model by using BT474 cells and the AGAP2-AS1 knockdown model by using SKBR-3 cells (Fig. 2a, b). The results from the MTT assay, revealed that BT474 cells overexpressed with AGAP2-AS1 showed significantly elevated levels of cell proliferation compared to negative controls, while knockdown of AGAP2-AS1 in SKBR-3 cells decreased cell proliferation (Fig. 2c). Further in the colony formation assay, the number of colonies formed was much higher in Lv-AGAP2-AS1-BT474 cells than Lv-NC-BT474 cells. However, a suppressed colony formation ability was identified in sh-AGAP2-AS1-SKBR-3 cells when compared to sh-NC-SKBR-3 cells (Fig. 2d). To confirm the effect of AGAP2-AS1 on cell growth, we investigated the Ki-67 expression level by immunofluorescence assay. As expected, an enhanced AGAP2-AS1 promoted Ki-67 expression was observed, whereas the AGAP2-AS1 knockdown dramatically silenced the level of Ki-67 (Fig. 2e). In addition, FACS apoptosis assay showed that overexpression of AGAP2-AS1 suppressed apoptosis whereas knockdown of AGAP2-AS1 exerted an opposite effect (Fig. 2f). To conclude, we demonstrated that AGAP2-AS1 played an oncogenic role in breast cancer.

**Fig. 2:** AGAP2-AS1 promotes proliferation and suppresses apoptosis of breast cancer cells. **a** The oligonucleotides labeled with GFP green fluorescence were transfected as described in the methods. **b** Transfection efficiency was identified by detecting AGAP2-AS1 expression via RT-qPCR. **c** MTT assay showed the functional effect of AGAP2-AS1 on cell proliferation of breast cancer cells. **d** Colony formation assay was used to determine the functional role of AGAP2-AS1. **e** Immunofluorescence analysis of Ki-67 expression in breast cancer cells after infection with respective oligonucleotides. **f** FACS apoptosis analysis of cells with overexpression or knockdown of AGAP2-AS1. **g, h** Cell viability was evaluated in cells treated with trastuzumab (0.5 mg/mL) after infection of respective oligonucleotides. **i** TUNEL assay was used to determine the function of AGAP2-AS1 for trastuzumab-induced cell apoptosis. *p < 0.05, **p < 0.01, ***p < 0.001

We also investigated whether AGAP2-AS1 regulates trastuzumab resistance. As expected, knockdown of AGAP2-AS1 promoted the trastuzumab-induced (0.5 μg/mL) cell cytotoxicity in the SKBR-3/Tr cells (Fig. 2g). In addition, overexpression of AGAP2-AS1 partially abrogated the effects of trastuzumab on cell viability in the BT474 parental cells (Fig. 2h). The TUNEL assay was then performed to analyze whether AGAP2-AS1 influenced the nuclear apoptosis induced by trastuzumab. We found that the overexpression of AGAP2-AS1 suppressed the trastuzumab-induced cell apoptosis in the BT474 parental cells whereas knockdown of AGAP2-AS1 enhanced the apoptosis caused by trastuzumab in the SKBR-3/Tr cells (Fig. 2i).

The article "SP1-induced lncRNA AGAP2-AS1 expression promotes chemoresistance of breast cancer by epigenetic regulation of MyD88" was retracted in 2023. Reasons: duplicated images; signs of a paper mill; unreliable results or conclusions.

### MyD88 is a downstream target of AGAP2-AS1 function in breast cancer cells

Based on the understanding of the pathologic role of AGAP2-AS1, we continued to explore the underlying regulatory mechanisms. RNA-pull down experiments were performed to search for the AGAP2-AS1-associated downstream proteins, and we found that MyD88 was enriched (Fig. 3a). MyD88 is an adaptor molecule for toll-like receptor (TLR) and interleukin 1 receptor (IL-1R) signaling implicated in tumorigenesis and resistance to chemotherapeutic drugs through proinflammatory mechanisms (Fig. 3b). Therefore, we assume that MyD88 could be important for trastuzumab resistance. In this study, we verified that the overexpression of AGAP2-AS1 upregulated the expression of MyD88 at both mRNA and protein levels (Fig. 3c), whereas knockdown of AGAP2-AS1 downregulated its expression (Fig. 3d). In addition, MyD88 was also upregulated in the trastuzumab-resistant cells when compared to their respective parental cells (Fig. 3e), strongly indicating that MyD88 may serve as a direct target of AGAP2-AS1.

**Fig. 3:** MyD88 is a downstream target of AGAP2-AS1 function in breast cancer. **a** RNA pull-down assay was performed to verify the enrichment of MyD88 by AGAP2-AS1 in the breast cancer cells. **b** Schematic diagram of the network of MyD88 based on ENCODE database (http://genome.ucsc.edu). **c**, **d** MyD88 was positively regulated by AGAP2-AS1 at both transcript and protein levels in SKBR-3 and BT474 cells. **e** MyD88 expression was determined in the trastuzumab-resistant and the parental breast cancer cells by western blot experiment. **f** MyD88 expression was detected via western blot after transfection of sh-MyD88 or Lv-MyD88. **g** Knockdown of MyD88 dramatically abrogated the effects of Lv-AGAP2-AS1 on cell proliferation whereas overexpression of MyD88 reversed the effect induced by sh-AGAP2-AS1. **h** Co-transfection of Lv-MyD88 reversed the effects of AGAP2-AS1 knockdown in SKBR-3/Tr cells whereas co-expression of sh-MyD88 abrogated the resistance induced by Lv-AGAP2-AS1 in the BT474 parental cells. *p < 0.05

To investigate whether MyD88 is a functional target of AGAP2-AS1, we constructed MyD88-overexpression vector and MyD88-knockdown vector (Fig. 3f). Then, we modulated the expression of endogenous AGAP2-AS1 and MyD88 simultaneously. The MTT assay revealed that silencing MyD88 significantly abrogated the effects of Lv-AGAP2-AS1 on cell growth, while overexpression of MyD88 reversed the effect induced by sh-AGAP2-AS1 (Fig. 3g). More importantly, Lv-MyD88 abrogated the sh-AGAP2-AS1-induced trastuzumab response in the SKBR-3/Tr cells whereas co-transfection of sh-MyD88 reversed the trastuzumab resistance induced by Lv-AGAP2-AS1 in the BT474 parental cells (Fig. 3h). Taken together, the lncRNA AGAP2-AS1 may promote trastuzumab resistance via binding to MyD88.

The article "SP1-induced lncRNA AGAP2-AS1 expression promotes chemoresistance of breast cancer by epigenetic regulation of MyD88" was retracted in 2023. Reasons: duplicated images; signs of a paper mill; unreliable results or conclusions.

### LncRNA AGAP2-AS1 induces an upregulation of MyD88 by modulating H3K27 acetylation

To further understand the regulation of MyD88 by AGAP2-AS1, we explored the probable mechanisms by analysis of the ENCODE database (http://genome.ucsc.edu/). As shown in Fig. 4a, there is a high concentration of H3K27ac in the promoter region of MyD88, indicating that MyD88 may be regulated at the transcriptional level via histone modification. To test this hypothesis, we performed a ChIP assay by using breast cancer parental and trastuzumab-resistant cells. As shown in Fig. 4b, an increased enrichment of H3K27ac was verified in breast cancer cells compared to normal cells. Moreover, an increased enrichment of H3K27ac was also verified in trastuzumab-resistant cells in contrast to the parental cells (Fig. 4c). We next treated breast cancer cells with C646, a histone acetyltransferase (HAT) inhibitor, and found a significant reduction in the MyD88 expression in response to the treatment (Fig. 4d). To this end, we demonstrated that MyD88 was upregulated in breast cancer cells due to the histone acetylation in its promoter region.

The article "SP1-induced lncRNA AGAP2-AS1 expression promotes chemoresistance of breast cancer by epigenetic regulation of MyD88" was retracted in 2023. Reasons: duplicated images; signs of a paper mill; unreliable results or conclusions.

**Fig. 4:** AGAP2-AS1 promotes the expression of MyD88 by modifying H3K27 acetylation. **a** Bioinformatics analysis showed that the promoter of MyD88 had a high enrichment of H3K27ac. **b** ChIP assay was used to verify the enrichment of H3K27ac in MyD88 promoter in the breast cancer cells and the normal breast epithelial cells. **c** ChIP assay showed that the enrichment of H3K27ac was higher in the trastuzumab resistant cells than in the parental cells. **d** MyD88 expression was detected by western blot in breast cancer cells treated with C646 or DMSO. **e** FISH analysis of the subcellular location of AGAP2-AS1 with a specific probe in breast cancer cells. **f** ChIP assay showed that AGAP2-AS1 positively regulated the enrichment of H3K27ac at the MyD88 promoter. *p < 0.05, ***p < 0.001

To further investigate whether lncRNA AGAP2-AS1 participates in the H3K27 acetylation at the MyD88 promoter, we identified the cellular localization of AGAP2-AS1 in breast cancer cells. FISH assay with a specific probe of AGAP2-AS1 confirmed that AGAP2-AS1 was mainly distributed in the nuclear section of both cells (Fig. 4e). Then, we detected whether AGAP2-AS1 regulates the enrichment of H3K27ac at the promoter region of MyD88. As expected, upregulation of AGAP2-AS1 in the BT474 cells increased the enrichment of H3K27ac whereas knockdown of AGAP2-AS1 resulted in a decrease in H3K27ac enrichment in the SKBR-3 cells (Fig. 4f). Therefore, we conclude that the lncRNA AGAP2-AS1 regulates MyD88 expression via the histone H3K27 acetylation.

### LncRNA AGAP2-AS1 mediates H3K27 acetylation at the promoter of MyD88 by binding with CBP

As CREB-binding protein (CBP) is an important enzyme that participates in chromatin acetylation, we explored whether CBP is essential for the AGAP2-AS1-regulated H3K27 acetylation of MyD88. As expected, overexpression of CBP using specific plasmids (Fig. 5a) dramatically increased the expression of MyD88 at both transcript and protein levels (Fig. 5b). The ChIP analysis showed that CBP was enriched at the MyD88 promoter regions (Fig. 5c), indicating that CBP may be essential for histone acetylation. On account of the above result that both AGAP2-AS1 and CBP could regulate H3K27 acetylation at the promoter of MyD88, we then tested whether AGAP2-AS1 and CBP are functionally linked during the histone acetylation process. We detected the CBP expression after knockdown or overexpression of AGAP2-AS1 and found that AGAP2-AS1 did not affect the expression level of CBP (Fig. 5d), so we hypothesized that AGAP2-AS1 may exert the oncogenic function by recruiting CBP to target genes. To test this assumption, we conducted RIP assay. As shown in Fig. 5e, an enriched AGAP2-AS1 was identified by anti-CBP antibody in contrast to anti-IgG. More importantly, AGAP2-AS1 influenced the enrichment of CBP and H3K27ac in the MyD88 promoter region (Fig. 5f, g). These results indicate that the binding of AGAP2-AS1 with CBP promoted the enrichment of H3K27ac, thereby resulting in the activation of MyD88 transcription.

The article "SP1-induced lncRNA AGAP2-AS1 expression promotes chemoresistance of breast cancer by epigenetic regulation of MyD88" was retracted in 2023. Reasons: duplicated images; signs of a paper mill; unreliable results or conclusions.

**Fig. 5:** AGAP2-AS1 mediates H3K27 acetylation at the promoter of MyD88 by binding with CBP. **a** CBP expression was detected by RT-qPCR. **b** The influence of CBP on MyD88 expression was identified by RT-qPCR (left panel) and western blot (right panel). **c** ChIP assay by using CBP antibody tested the enrichment at MyD88 promoter. **d** Western blot analysis indicated that AGAP2-AS1 showed little effect on CBP expression. **e** RIP experiment showed that anti-CBP antibody could precipitate AGAP2-AS1 in SKBR-3 and BT474 cells. **f**, **g** ChIP-qPCR revealed that AGAP2-AS1 influenced the enrichment of CBP and the level of H3K27ac acetylation at the promoter region of MyD88. *p < 0.05, **p < 0.01, ***p < 0.001

### LncRNA AGAP2-AS1 facilitates tumor growth and trastuzumab resistance via MyD88 in vivo

To validate the in vitro data of lncRNA AGAP2-AS1, we established a model of nude mice bearing the BT474 xenograft. The BT474 cells infected with Lv-AGAP2-AS1 or Lv-NC were planted into the flanks of nude mice. Four treatment groups of mice xenograft were established: Group I (Lv-NC-transfected cells + PBS), Group II (Lv-AGAP2-AS1-transfected cells + PBS), Group III (Lv-NC-transfected cells + trastuzumab treatment) and Group IV (Lv- AGAP2-AS1-transfected cells + trastuzumab treatment). Then, tumors were stripped and presented as in Fig. 6a. The results showed that AGAP2-AS1 promoted tumor growth in xenograft model (Group II vs. Group I). Trastuzumab treatment significantly suppressed the growth of tumor cells when compared to the control groups (Group III vs. Group I). With the treatment of trastuzumab, the tumor cells that were infected with Lv-AGAP2-AS1 grew faster than Lv-NC-transfected cells (Group IV vs. Group III), suggesting that AGAP2-AS1 promoted trastuzumab resistance in vivo (Fig. 6b).

**Fig. 6:** AGAP2-AS1 facilitates trastuzumab resistance via MyD88 in vivo*.* **a** Images of tumors that developed in xenograft transplanted nude mouse tumor models treated by administering 5 mg/kg trastuzumab or PBS (for control group) intraperitoneally once every 2 days for 3 weeks in different groups. Four treatment groups of mice xenograft were established: Group I (Lv-NC-transfected cells + PBS), Group II (Lv-AGAP2-AS1-transfected cells + PBS), Group III (Lv-NC-transfected cells + trastuzumab treatment) and Group IV (Lv- AGAP2-AS1-transfected cells + trastuzumab treatment). Six mice were included in each group and more than three mice remained after the treatment regimen excluding mice that were dead or with complications, such as skin necrosis due to infection. **b** Weights of tumors that developed in xenografts from different groups are shown. **c** IHC analysis of expression levels of MyD88 in respective groups. **d** Images of tumors that developed in xenograft transplanted nude mouse tumor models treated orally with 5 mg/kg gefitinib once daily for 3 weeks in different transfection groups. *p < 0.05, **p < 0.01

In addition, IHC experiment was conducted to verify whether AGAP2-AS1 affects the expression of MyD88 in xenograft tumor tissues. As shown in Fig. 6c, overexpression of AGAP2-AS1 promoted the expression of MyD88 in tumor tissues (Group II vs. Group I, or Group IV vs. Group III, respectively), indicating that AGAP2-AS1 regulates tumor growth and trastuzumab resistance via targeting MyD88 in vivo. To directly verify whether MyD88 could rescue the effects of AGAP2-AS1 in vivo, we injected the BT474 cells that were co-transfected with sh-MyD88 and Lv-AGAP2-AS1 followed by trastuzumab treatment as described above. As expected, co-transfection of sh-MyD88 dramatically reversed the Lv-AGAP2-AS1-induced trastuzumab resistance in vivo (Fig. 6d), further confirming that MyD88 is essential for the carcinogenic function of AGAP2-AS1.

The article "SP1-induced lncRNA AGAP2-AS1 expression promotes chemoresistance of breast cancer by epigenetic regulation of MyD88" was retracted in 2023. Reasons: duplicated images; signs of a paper mill; unreliable results or conclusions.

### NF-κB signaling pathway is activated by the overexpression of Myd88 induced by AGAP2-AS1

There is sufficient evidence indicating that MyD88 regulates cancer cell proliferation, apoptosis and chemoresistance by the activation of NF-κB pathway. As we have proved that lncRNA AGAP2-AS1 promotes trastuzumab resistance via enhancing MyD88 expression by modifying histone acetylation, we hypothesized that the NF-κB pathway may be involved in the oncogenic role of AGAP2-AS1 and MyD88. Western blot experiment was performed to test this hypothesis, and we found that NF-κB activity was suppressed in sh-AGAP2-AS1-SKBR-3 cells, while ectopic expression of MyD88 rescued this effect (Fig. 7a). Conversely, NF-κB activity increased in the BT474 cells transfected with Lv-AGAP2-AS1 compared to the negative control cells, while silencing of MyD88 diminished this enhanced activity induced by AGAP2-AS1 overexpression (Fig. 7b). To this end, we demonstrated that AGAP2-AS1 promoted tumor growth via upregulation of MyD88 expression and further activation of NF-κB signaling pathway.

**Fig. 7:** NF-κB signaling pathways is promoted by the upregulation of MyD88 induced by AGAP2-AS1. **a** Western blot was performed to detect the activity of NF-κB in AGAP2-AS1-silenced SKBR-3 cells transfected with Lv-MyD88. **b** Western blot was performed to detect the activity of NF-κB in AGAP2-AS1-overexpressing BT474 cells transfected with sh-MyD88

The article "SP1-induced lncRNA AGAP2-AS1 expression promotes chemoresistance of breast cancer by epigenetic regulation of MyD88" was retracted in 2023. Reasons: duplicated images; signs of a paper mill; unreliable results or conclusions.

### AGAP2-AS1 expression is associated with the response to trastuzumab therapy in patients with breast cancer

We detected the expression of AGAP2-AS1 in 42 breast cancer tissues and paired adjacent non-tumor tissues. As shown in Fig. 8a, AGAP2-AS1 expression frequently increased in cancerous tissues and 69% of the cancer samples displayed increased AGAP2-AS1 expression in our study. MyD88 was upregulated in 76.2% of breast cancer patients. In addition, correlation analysis by using Spearman testing confirmed a significant positive correlation between the expression of AGAP2-AS1 and MyD88 in these specimens (Fig. 8b).

**Fig. 8:** AGAP2-AS1 expression is associated with chemoresponse to trastuzumab therapy in patients with breast cancer. **a** The expressions of AGAP2-AS1 and MyD88 in 42 paired breast cancer tissues. **b** The statistically significant association between AGAP2-AS1 and MyD88 expression in breast cancer specimens. **c** AGAP2-AS1 expression was determined via RT-qPCR for the trastuzumab-resistant and sensitive patients. **d** ROC curve was established to show the ability of AGAP2-AS1 in differentiating responding patients from non-responding patients. **e** The proportion of patients that showed resistance to trastuzumab therapy was significantly higher in high AGAP2-AS1 expressing groups than in low expression group. ***p < 0.001

To verify the clinical role of AGAP2-AS1 in trastuzumab-treated patients, we collected 62 cancer tissues from advanced HER2^+^ breast cancer patients who received trastuzumab treatment. Patients were divided into responding (CR + PR, 33 patients) and non-responding (SD + PD, 29 patients) groups according to the immuno-related Response Evaluation Criteria In Solid Tumors (irRECIST) [20]. RT-qPCR revealed that AGAP2-AS1 was upregulated in the non-responding group (Fig. 8c). We then investigated the value of AGAP2-AS1 in differentiating responding patients from non-responding patients by establishing ROC curve. As shown in Fig. 8d, the area under the curve (AUC), diagnostic sensitivity, and specificity reached 0.753, 78.7 and 63.7% with the established cut-offs (3.78), respectively. Under this stratification criteria (3.78), patients were divided into a low and a high AGAP2-AS1 expression groups, and the proportion of patients not responding to chemotherapy was significantly higher in the high AGAP2-AS1 expression group than in the low expression group (Fig. 8e). Altogether, our clinical results indicate that AGAP2-AS1 may be a promising prognostic marker to discriminate responders and non-responders to trastuzumab therapy.

The article "SP1-induced lncRNA AGAP2-AS1 expression promotes chemoresistance of breast cancer by epigenetic regulation of MyD88" was retracted in 2023. Reasons: duplicated images; signs of a paper mill; unreliable results or conclusions.

## Discussion

Extensive efforts in the past have contributed to the understanding of both molecular and cellular mechanisms of action of chemo-resistance, one of the major causes for the failure of treatment of advanced cancer types. However, little progress has been made ever since [21]. Thus, the discovery of novel molecular signatures seems to hold a great promise in tumor characterization and could be used as a potential therapeutic target. To identify potential molecular biomarkers for trastuzumab treatment; the functional relevance of lncRNA AGAP2-AS1 expression with trastuzumab resistance in breast cancer was investigated. Our results indicated that AGAP2-AS1 regulated tumor growth, apoptosis, and chemo-resistance via upregulation of MyD88 expression through binding with CBP and modifying H3K27 acetylation (Fig. 9).

**Fig. 9:** A schematic diagram representing the role of AGAP2-AS1 in breast cancer chemoresistance via upregulating MyD88 expression through modifying H3K27 acetylation

It is well known that breast cancer patients overexpressing HER2 are associated with poor prognosis [22]. HER2 gene amplification was first associated with worse clinical outcomes in the late 1980s by Slamon et al., and the following series of studies revealed that residents of the Asia-Pacific areas were associated with high occurrence rate HER2-positive cancer with a poorer prognosis in comparison with other regions [23–25]. Although trastuzumab remains the standard treatment for patients with HER2 overexpressing breast cancer in neoadjuvant, adjuvant and metastatic settings, the presence of acquired and de novo resistance is a serious concern. The understanding of resistance mechanisms could allow developing strategies to prevent and/or overcome this resistance [26].

LncRNA AGAP2-AS1 was recently verified as an oncogene in NSCLC and gastric cancer [13, 19, 27], but the expression in breast cancer is not reported. In this study, we identified the expression level of AGAP2-AS1 and investigated its functional role in breast cancer. Consistent with previous reports, our results showed that AGAP2-AS1 was upregulated in breast cancer and promoted tumor growth and chemoresistance to trastuzumab. To further investigate the regulatory mechanism by which AGAP2-AS1 plays an oncogenic role, we determined the down-stream target genes by conducting RNA-pull down experiments. On this basis, we identified MyD88, which has an N-terminal death domain (DD), which recruits downstream signaling molecules [28]. MyD88 and TLR4 specific binding plays an important biological function in pathogenesis by mediating tumor invasion and migration, escaping from immunosurveillence, promoting tumor proliferation, inhibiting apoptosis, and developing chemoresistance in cancer [29–31]. Egunsola et al. reported that silencing of MyD88 expression could effectively reduce lung metastasis in breast cancer mouse model as well as decrease CCL2 and CCL5 expression [32]. Our study showed that MyD88 is upregulated by AGAP2-AS1 and is essential for the functioning of AGAP2-AS1, suggesting that AGAP2-AS1 regulates trastuzumab resistance via targeting MyD88.

The article "SP1-induced lncRNA AGAP2-AS1 expression promotes chemoresistance of breast cancer by epigenetic regulation of MyD88" was retracted in 2023. Reasons: duplicated images; signs of a paper mill; unreliable results or conclusions.

The mechanisms that generate transcript diversity are of fundamental importance in cancers. In recent years, the epigenetic factors such as chromatin modifications, have not only been implicated in the spatio-temporal regulation of gene expression, but also influences how these transcripts are processed [33]. In addition, many studies revealed that lncRNAs could play an important role in regulating gene expression by epigenetic modifications [34, 35]. AGAP2-AS1 could bind to the promoter regions of targeted genes and influence their transcriptions [13]. Hence, we tested whether AGAP2-AS1 could regulate genes by epigenetic modifications. In this study, bioinformatics analysis using the ENCODE database, followed by ChIP assay showed that H3K27ac was highly enriched at the promoter of MyD88, and this histone acetylation was mediated by AGAP2-AS1 as evidenced by the fact that the enrichment level was influenced by AGAP2-AS1 expression in the breast cancer cells. Histone acetylation is a major histone modification involved in the regulation of chromatin structure and transcription. It neutralizes the positive charge on the lysine side chain, relaxing the chromatin structure and enhancing transcriptional activity [36]. Herein, our study revealed the H3K27 modification at the MyD88 promoter region by AGAP2-AS1 in breast cancer cells.

Recent evidences suggest that lncRNAs could serve as scaffolds for chromatin-modifying complexes and act as signals in response to DNA damage, suggesting that the regulatory function of lncRNAs is dependent on its interacting proteins [37]. CBP is a transcriptional co-activator with histone acetyltransferase (HAT) activity that was shown to be important for histone acetylation [38, 39]. More recently, a profile of RNAs was reported to bind with CBP to influence gene expression through modifying histone acetylation [40]. In this study, we verified that AGAP2-AS1 could interact with CBP to form an active complex, which upregulated MyD88 expression via promoting the enrichment of H3K27ac at the promoter region of MyD88, further activating the NF-κB signaling pathway.

The article "SP1-induced lncRNA AGAP2-AS1 expression promotes chemoresistance of breast cancer by epigenetic regulation of MyD88" was retracted in 2023. Reasons: duplicated images; signs of a paper mill; unreliable results or conclusions.

Finally, we explored the potential translational applications of AGAP2-AS1 in breast cancer patients. By performing ROC curve analysis, we identified that AGAP2-AS1 showed a relatively high prognostic value when using it for discriminating responders and non-responders to trastuzumab therapy. However, further studies are warranted before lncRNAs like AGAP2-AS1 could be used for clinical applications. In addition, the prognostic influence of AGAP2-AS1 on survival of breast cancer patients needs to be further investigated.

## Conclusion

Our study demonstrated that the lncRNA AGAP2-AS1 promotes oncogenesis and chemoresistance to trastuzumab treatment of breast cancer via regulating MyD88*.* Therefore, AGAP2-AS1 may be a promising therapeutic target for breast cancer patients, enhancing the clinical benefits of trastuzumab therapy.

## Additional file

Additional file 1: **Table S1.** Information of the qPCR primer sequences and siRNA sequences. (DOC 35 kb)

## Abbreviations

AUC: Area under the curve
CBP: CREB-binding protein;
ChIP: Chromatin immunoprecipitation
DAPI: 4′,6-diamidino-2-phenylindole
DMEM: Dulbecco’s modified Eagle’s medium
FBS: Fetal bovine serum
FISH: Fluorescence in situ hybridization
GAPDH: Glyceraldehyde 3-phosphate dehydrogenase
HAT: Histone acetyltransferase;
HER2: Human epidermal growth factor receptor 2
IHC: Immunochemistry
lncRNA: Long Noncoding RNA
MyD88: Myeloid differentiation factor 88
NC: Negative control
PCR: Polymerase chain reaction
RIP: RNA immunoprecipitation
ROC: Receiver operating characteristic
SD: Standard deviation
TFs: Transcription factors
